RETRACTED

# HIF-1α Affects the Neural Stem Cell Differentiation of Human Induced Pluripotent Stem Cells via MFN2-Mediated Wnt/β-Catenin Signaling

**DOI:** 10.3389/fcell.2021.671704

**Published:** 2021-06-21

**Authors:** Peng Cui, Ping Zhang, Lin Yuan, Li Wang, Xin Guo, Guanghui Cui, Yanmin Zhang, Minghua Li, Xiaowei Zhang, Xiaoqiang Li, Yuxin Yin, Zhendong Yu

**Affiliations:** ^1^Institute of Precision of Medicine, Peking University Shenzhen Hospital, Shenzhen, China; ^2^Department of Hematology, Peking University Shenzhen Hospital, Shenzhen, China; ^3^Department of Biochemistry, University of Texas Southwestern Medical Center, Dallas, TX, United States; ^4^Department of Oncology, Peking University Shenzhen Hospital, Shenzhen, China; ^5^Central Laboratory, Peking University Shenzhen Hospital, Shenzhen, China; ^6^School of Basic Medical Sciences, Peking University, Beijing, China; ^7^Department of Thoracic Surgery, Peking University Shenzhen Hospital, Shenzhen, China; ^8^Institute of Systems Biomedicine, Department of Pathology, School of Basic Medical Sciences, Peking-Tsinghua Center for Life Sciences, Peking University Health Science Center, Beijing, China

**Keywords:** induced pluripotent stem cells, hypoxia-inducible factor 1α, mitofusin2, differentiation, neural stem cells

## Abstract

Hypoxia-inducible factor 1α (HIF-1α) plays pivotal roles in maintaining pluripotency, and the developmental potential of pluripotent stem cells (PSCs). However, the mechanisms underlying HIF-1α regulation of neural stem cell (NSC) differentiation of human induced pluripotent stem cells (hiPSCs) remains unclear. In this study, we demonstrated that HIF-1α knockdown significantly inhibits the pluripotency and self-renewal potential of hiPSCs. We further uncovered that the disruption of HIF-1α promotes the NSC differentiation and development potential *in vitro* and *in vivo*. Mechanistically, HIF-1α knockdown significantly enhances mitofusin2 (MFN2)-mediated Wnt/β-catenin signaling, and excessive mitochondrial fusion could also promote the NSC differentiation potential of hiPSCs via activating the β-catenin signaling. Additionally, MFN2 significantly reverses the effects of HIF-1α overexpression on the NSC differentiation potential and β-catenin activity of hiPSCs. Furthermore, Wnt/β-catenin signaling inhibition could also reverse the effects of HIF-1α knockdown on the NSC differentiation potential of hiPSCs. This study provided a novel strategy for improving the directed differentiation efficiency of functional NSCs. These findings are important for the development of potential clinical interventions for neurological diseases caused by metabolic disorders.

## Introduction

Pluripotent stem cells (PSCs) undergo unlimited self-renewal and hold the potential to differentiate into various cell types in the three germ layers (Ying et al., 2008; Ding et al., 2015). Terminally differentiated somatic cells and adult stem cells (ASCs) can be reprogrammed into induced pluripotent stem cells (iPSCs) via the classic “Yamanaka factors” transfection (Takahashi and Yamanaka, 2006), thus providing new hope for the development of regenerative medicine and patient-refractory cell therapy (Gintant et al., 2017; Nakajima et al., 2018; Blau and Daley, 2019; Rowe and Daley, 2019). During the pluripotency maintenance, differentiation, and reprogramming of iPSCs, transcription factors, epigenetic modifications, mitochondrial characteristics, and metabolic pattern transitions play a vital role (Pan and Thomson, 2007; Wang T. et al., 2011; Guo et al., 2017). Stem cells with different pluripotency tend to use different metabolic pathways to maintain their normal life activities. To some extent, PSCs, including embryonic stem cells, iPSCs, and ASCs, possess high glycolytic activity to meet the adenosine-triphosphate (ATP) requirements, whereas terminally differentiated cells rely on oxidative phosphorylation (OXPHOS) for energy metabolism (Wanet et al., 2015). Recent studies have indicated that the different metabolic patterns of PSCs are closely related to self-renewal and the initial cell fate decision, and during differentiation into somatic cells, the metabolic patterns change from aerobic glycolysis to OXPHOS (Teslaa and Teitell, 2015). However, the changes in metabolic and regulatory mechanisms involved in human induced pluripotent stem cell (hiPSC) differentiation into ASCs, such as neural stem cells (NSCs), remain unclear.

RETRACTED

Hypoxia is vital to maintain the cell metabolic balance and embryonic development (Mohyeldin et al., 2010), and is considered a key feature of the stem cell niche (Suda et al., 2011), and is beneficial for hiPSCs and ASCs (Ezashi et al., 2005; Simsek et al., 2010; Stegen et al., 2019). Hypoxia-inducible factor 1α (HIF-1α) is an important transcription factor that allows stem cells to adapt to hypoxic environments and maintain pluripotency and developmental potential. Numerous reports have shown that HIF-1α activates genes involved in pluripotency and metabolism to maintain the functional transition of stem cells (Takubo et al., 2010; Mathieu et al., 2014; Wang Y. et al., 2011). Research into the regulatory mechanisms underlying HIF-1α activity in PSCs will thus provide new insight into stem cell biology under hypoxia.

Mitochondria exist in an equilibrium wherein their morphology is constantly altered to participate in cell metabolism, proliferation, differentiation, cell cycle, intracellular calcium balance, apoptosis, and aging (Li et al., 2017; Seo et al., 2018; Dong et al., 2020). The balance of mitochondrial dynamics depending on the chronological regulation of mitochondrial fusion and fission proteins plays extremely pivotal roles in tissue formation and embryonic development (Chen et al., 2003). Imbalances in mitochondrial dynamics lead to the disturbed development of NSCs during neurogenesis (Züchner et al., 2004; Misko et al., 2012). Clinically, the dysregulation of mitochondrial dynamics has also been closely linked to many neurological degenerative diseases, including Alzheimer disease (AD) and Parkinson disease (PD) (Deng et al., 2008; Yang et al., 2008; Burte et al., 2015). As a mitochondrial fusion protein, mitofusin2 (MFN2) knockdown results in mitochondrial functional network disorders, diabetic cardiomyopathy and sarcopenia (Sebastián et al., 2016; Hu et al., 2019), and hinders neuronal differentiation and synapse formation (Lee et al., 2012; Fang et al., 2016). Knowledge regarding the impact of mitochondrial dynamics on hiPSC function is limited. Some data show that mitochondrial morphology and bioenergetics undergo opposite and reversible conversions during hiPSC reprogramming and differentiation (Son et al., 2015; Wanet et al., 2015; Prieto et al., 2016). Recent studies have indicated that mouse iPSCs with different developmental potential express different levels of mitochondrial proteins, and the imbalance of mitochondrial dynamics seriously affects the differentiation and developmental potential of mouse iPSCs. Mitochondrial fission factor (MFF) affects the developmental potential of mouse iPSCs by regulating the calmodulin pathway-mediated ubiquitination degradation of β-catenin (Zhong et al., 2019).

RETRACTED

Whereas it has been established that mitochondrial metabolic disorders can affect the balance of mitochondrial dynamics, the molecular mechanism through which mitochondrial metabolism affects hiPSC differentiation into NSCs by regulating mitochondrial dynamics is unclear. In this study, we aimed to explore the effects of HIF-1α on hiPSC pluripotency, self-renewal, and metabolic potential, by investigating the mitochondrial membrane potential (ΔΨm) and intracellular reactive oxygen species (ROS). Moreover, we determined that HIF-1α knockdown promotes the NSC differentiation by enhancing MFN2-mediated β-catenin signaling. Meanwhile, MFN2 could further reverse the effects of HIF-1α on the NSC differentiation efficiency and β-catenin expression of hiPSCs. Moreover, Wnt/β-catenin signaling inhibition could reverse the effects of HIF-1α knockdown on the NSC differentiation potential of hiPSCs.

## Materials and Methods

### hiPSCs Culture

The hiPSCs were a gift from Guangzhou Institutes of Biomedicine and Health, Chinese Academy of Sciences, which were cultured in mTesR1 complete medium (85850, STEM CELL Technologies) on the diluted Matrigel (354277, Corning). In brief, primed hiPSCs were required to be replaced with fresh medium every days, and were subcultured to small monolayer clones once every 4 days by 0.5 mM ethylenediaminetetraacetic acid (EDTA) (15575020, Thermo Fisher Scientific) digestion in a 37°C incubator for 3 min.

### Establishment of Gene-Modified hiPSCs Cell Lines

Hypoxia-inducible factor 1α and MFN2 overexpression/short hairpin RNA (shRNA) plasmids were purchased from Hanbio Biotechnology. Resistance gene-linked overexpression or shRNA plasmids, pMD2.G and pSPAX2 lentiviral packaging plasmid were co-transfected into HEK293T cells using Lipofectamine^TM^ 3000 (L3000015, Thermo Fisher Scientific) in a ratio of 1: 2: 3. The culture supernatant containing virus particles was collected and slowly filtered into a virus ultrafiltration tube to concentrate the lentivirus at 48 and 72 h after transduction. hiPSCs with 30% confluence in logarithmic growth phase were infected with equal amounts of target and non-target control (NC) lentivirus with 6 mg/mL polybrene (sc-134220, Santa Cruz) in half the amount of medium. The medium was added to 2 ml in the six-well plate, and replaced by the fresh mTesR1 24 h after infection. The lentivirus-treated hiPSCs were screened with 10 μg/mL Blasticidin S (BSD; B9300, Solarbio) and 1 μg/mL Puromycin (PURO; ant-pr-5, Thermo Fisher Scientific) for positive viable cell line. After 2 weeks of screening, the overexpressed and knockdown hiPSCs were expanded, and verified the gene expression by quantitative RT-PCR (qRT-PCR) and western blot.

### Cell Proliferation Assay

Human induced pluripotent stem cells in logarithmic growth phase were digested into single cells with Accutase (A1110501, Thermo Fisher Scientific) in a 37°C incubator for 3 min, and were seeded into the Matrigel-coated 96-well plates at a density of 5000 cells per well. The assayed hiPSCs were cultured with complete mTesR1 medium mixed 10 μM ROCK inhibitor (Y27632; A1110501, STEM CELL Technologies) for the initial 24 h, and removed it after 24 h. The OD value reflecting cell proliferation was detected by fully automatic microplate reader (Thermo Fisher Scientific) after cell counting kit-8 (CCK8) (PA584814, Thermo Fisher Scientific) treatment for 4 h on day 1–5, respectively.

### Clonogenic Assay

Clonogenic assays of NC and genetically modified hiPSCs were performed in the state of single cell growth. 2000 single cells were seeded into a twelve-well plate with pre-coated Matrigel in mTeSR1 medium supplemented with 10 μM Y27632 on first day, and all the non-adherent dead cells were removed by changing into the fresh mTeSR1 medium without Y27632 on the next day. hiPSCs cultured for 7 days were stained with Alkaline Phosphatase (AP) Assay Kit (C3206, Beyotime), photographed and counted the number and sizes of colonies.

RETRACTED

### AP Staining

Human induced pluripotent stem cells were subcultured and fixed with 4% of (w/v) paraformaldehyde for 15 min at room temperature, and cells were rinsed with D-PBS for three times, and then incubated with BCIP/NBT at 37°C for 20 min in 37°C incubator. BCIP/NBT was removed and fresh D-PBS was added. The AP performance of hiPSCs was analyzed by confocal microscopy. For the detection of AP activity, 5 × 10^5^ cells were fully lysed by the cell lysis buffer, and were resuspended with 50 μL of D-PBS, and 50 μL of chromogenic substrate wad added into the cell suspension. The mixture was incubated at 37°C incubator for 15 min. The AP activity was detected by a microplate reader at the wavelength of 405 nm. AP staining and activity were performed using the Alkaline Phosphatase Assay Kit (C3206, Beyotime) according to the manufacturer’s protocol.

### Immunofluorescence Staining

Cell samples were fixed for 20 min in 4% (w/v) paraformaldehyde (0.01 mol/L, pH 7.4) (1.43904.0500, Merck Millipore) at room temperature (RT), and permeabilized with 0.1% Triton X-100 (V900502, Sigma) in D-PBS for 20 min at RT, and then blocked with 2% BSA (A1933, Sigma) for 1 h after washing with D-PBS for three 5 min, followed by incubating with primary antibodies, were purchased from CST, against MFN2 (1:100, 11925S, CST), β-catenin (1:100, 8480T, CST), Nestin (1:200, 33475S, CST), and PAX6 (1:3200, 60433S, CST) at 4°C overnight. On next day, cells were incubated with Alexa Fluor fluorescent tag-conjugated secondary antibodies diluted in 2% BSA for 1 h at RT after three 5 min washes in D-PBS. Nuclei were stained with 10 mg/mL Hoechst 33342 (DH164-1, Sigma) for 5 min at RT and protected from light. Cells were imaged by a laser scanning confocal microscope (Zeiss LSM 780) immediately after three washes with D-PBS.

### Measurement of Mitochondrial Membrane Potential (ΔΨm)

The cationic fluorescent dye tetramethylrhodamine methyl ester (TMRE) (HY-D985A, MCE), as a mitochondrial probe, was used for monitoring the mitochondrial ΔΨm in living cells. TMRE was diluted with DMSO (0.5 mM stock solution) and added to the mTesR1 medium with a final concentration of 50 nM. hiPSCs were rinsed with D-PBS for three 5 min and then incubated with TMRE working solution at 37°C for 20 min, TMRE was removed and rinsed with D-PBS the fresh mTesR1 complete medium was supplemented. ΔΨm of hiPSCs was analyzed by confocal microscopy and flow cytometry immediately.

RETRACTED

### Measurement of ROS

MitoSox Red (40778ES50, YEASEN), as a fluorogenic dye for the highly selective detection of superoxide in mitochondria, was used to measure the mitochondrial ROS production of hiPSCs. hiPSCs were rinsed with D-PBS and incubated with 5 mM MitoSox Red for 20 min at 37°C. Nuclei were stained with 10 mg/mL Hoechst 33342 for 5 min in the dark after three washes with D-PBS, and the ROS production of hiPSCs was analyzed by confocal microscopy. Additionally, intracellular oxidative stress of hiPSCs was determined based on the oxidation of 2′,7′-dichlorodihydrofluorescein diacetate (DCFH-DA) (AAT-15204, AAT Bioquest). Cells were treated similarly to MitoSox Red staining assays, and incubated with 10 mM DCFH-DA for 30 min at RT. After the dyes were loaded, hiPSCs were digested and collected to analyze the ROS production by flow cytometry.

### Determination of ATP Levels

Intracellular ATP levels were measured by the ATP assay kit (AAT-15204, Abnova). 1 × 10^4^ hiPSCs were seeded in white opaque microplates. After 24 h, the culture medium was removed and changed into the Reconstituted Reagent (95 μL Assay Buffer with 1 μL Substrate and 1 μL ATP enzyme); 90 μL of Reconstituted Reagent was added to each well, and ATP production was measured on a Luminometer (Promage) within 1 min.

### Quantitative RT-PCR (qRT-PCR)

Quantitative RT-PCR was performed as previously described (Zhong et al., 2019). Total RNA was isolated using Trizol reagent (15596026, Thermo Fisher Scientific), and then RNA was reverse transcribed to cDNA using Evo M-MLV RT Kit with gDNA Clean (15596026, Accurate Biotechnology). qRT-PCR was performed using SYBR^®^ Green Premix Pro Taq HS qPCR Kit (AG11701, Accurate Biotechnology) on the iCycler Real-time System (Bio-Rad). The reaction conditions were 95°C for 3 min, followed by 45 cycles at 95°C for 30 s and 60°C for 30 s. All reactions were run in triplicates and the details of primers are listed in Supplementary Table.

### Western Blot Analysis

Western blot was performed according to the previous study (Zhong et al., 2019). Monoclonal Primary antibodies at the different dilutions were used as follows: HIF-1α (1:1000, 610958, BD), Nanog (1:1000, 3580S, CST), OCT4 (1:1000, 2750S, CST), MFN2 (1:1000, 11925S, CST), WNT3a (1:1000, A0642, ABclonal Technology), WNT5a (1:1000, A19133, ABclonal Technology), GSK-3ɑ(1:1000, A19060, ABclonal Technology), GSK-3β (1:1000, A11731, ABclonal Technology), β-catenin (1:1000, 8480T, CST), β-actin (1:1000, 4967L, CST), and COX IV (1:1000, 4850T, CST).

RETRACTED

### Embryoid Body (EB) Formation Assay

Embryoid body (EB) formation assay was performed according to the previous study (Zhang et al., 2018). hiPSCs in the logarithmic growth phase were rinsed once with D-PBS, and then digested into large clones with 1 mg/mL dispase II (D4693, Sigma) for 15 min in a 37°C incubator. Cells were collected and centrifuged by low-speed centrifugation at 500 rpm for 3 min. After rinsing with DF12 and centrifugation, the supernatant was removed and the clone masses were resuspended in EB medium supplemented with 10 μM Y27632 by a 5 ml pipette, and inoculated into low-adherent cell culture dishes. Y27632 was added into the EB medium for the first 24 h to ensure a high survival rate of the cells. EB medium was changed every other day by natural precipitation in a 37°C incubator, and EBs samples were collected on day 2, 4, and 6.

### Teratoma Formation Assay

For teratoma formation of hiPSCs in immunodeficient mice, 3 × 10^6^ hiPSCs were harvested according to the method of EB formation assay. Finally, the cell masses were rinsed with D-PBS and suspended in D-PBS with 30% Matrigel, and then 100 μL cell suspension was subcutaneously injected into each hind leg of the severe combined immunodeficiency (SCID) mice of 5–6 weeks old under a sterile stereo microscope. The teratomas were recovered 40 days after transplantation. About 40 days later, the SCID mice were euthanized and the teratomas were weighed, fixed, sliced, and stained using monoclonal antibodies (Nestin and PAX6) of NSCs, and stained with hematoxylin and eosin (H&E) for histological analysis. Teratomas were examined following the guidelines and regulations of the Institutional Animal Care and Use Committee (IACUC).

### Mito Tracker Staining

Human induced pluripotent stem cells were seeded on Matrigel-coated coverslips. As the cells proliferated to the logarithmic growth phase after 2 days, the cells were incubated with a pre-warmed staining working solution containing 50 nM MitoTracker Green (C1048, Beyotime) at 37°C for 30 min. After rinsing with D-PBS, cells were fixed with 4% paraformaldehyde (PFA) and stained with 10 mg/mL Hoechst 33342 for 5 min in the dark. Images were analyzed by confocal microscopy. The acquisition and assessment of images were performed in random order using ZEN microscope imaging software.

### EB-Derived NSC Differentiation

About 500 EBs spontaneously differentiated on day 6 were inoculated into Matrigel-plated six-well plates at a suitable density. On the next day, EB medium was replaced with NSC pre-differentiation medium supplemented with 20 ng/ml basic fibroblast growth factor (bFGF) (AF-100-18C, Peprotech). The medium was changed every other day. In the third generation, cell medium was changed to the completed differentiation medium supplemented with 20 ng/ml bFGF and 20 ng/ml epidermal growth factor (EGF) (AF-100-15, Peprotech). When obvious rosettes appeared in the culture dish, cells were collected for NSC markers identification by immunofluorescence staining.

RETRACTED

### Small Molecules Induced NSC Differentiation

Small molecules induced NSC differentiation was performed using the protocol from Dr. Ding (Li et al., 2011). hiPSCs at about 30% confluence were treated with 2 μM SB431542 (72232, STEM CELL Technologies), 3 μM CHIR99021 (HY-10182, MCE), 0.1 μM Compound E (HY-14176, MCE) in NSC differentiation induction media containing DMEM/F12:Neurobasal (1:1), 1 × N2 (17508-048, Thermo Fisher Scientific),1 × B27 (17504044, Thermo Fisher Scientific), 1% Glutmax, 5 μg/mL BSA and 10 ng/mL hLIF (8911, CST), for 7 days. Pre-induced hiPSCs were split 1:3 for the next three passages using Accutase and then replaced with NSC differentiation induction media supplemented with 2 μM SB431542 and 3 μM CHIR99021 on Matrigel-coated plates. After six passages, the NSCs were split 1:10 every 5 days. NSCs after two-step induction were collected for NSC markers identification by immunofluorescence staining. During the initial few passages, 10 μM Y27632 was required to supplement to enhance cell survival.

### Statistical Analysis

Throughout the paper, *p* values were calculated with Student’s *t* test. ^∗^*p* < 0.05, ^∗∗^*p* < 0.01, ^∗∗∗^*p* < 0.001 vs. hiPSCs (CON) or HIF-1α NC hiPSCs or MFN2 NC hiPSCs, and ^#^*p* < 0.05, ^##^*p* < 0.01, ^###^*p* < 0.001 vs. HIF-1α OE hiPSCs or HIF-1α sh hiPSCs. Scale bars show the SEM of at least three separate experiments.

## Results

### HIF-1α Regulates hiPSC Mitochondrial Metabolism and Dynamics

As described previously, HIF-1α knockdown significantly decreased AP activity, self-renewal ability and mitochondrial metabolic performance of hiPSCs (Cui et al., 2020). Next, we also detected the effects of HIF-1α on proliferation ability of hiPSCs using clonogenic assays. The results further revealed that HIF-1α knockdown significantly inhibited the colony formation ability and the self-renewal ability of hiPSCs (Figure 1A). Additionally, the expression of glycolytic and OXPHOS markers, such as lactate dehydrogenase A (LDHA) and Cytochrome c oxidase subunit 7a1 (COX7a1), was examined, and the results showed that HIF-1α knockdown significantly reduced glycolytic activity and significantly increased the OXPHOS activity in hiPSCs (Figure 1B).

**FIGURE 1:** Hypoxia-inducible factor 1α (HIF-1α) regulates hiPSC pluripotency self-renewal and mitochondrial dynamics. **(A)** Clonogenic assays, formation efficiency and colony diameter statistics of HIF-1α-modified hiPSCs. Scale bars, 100 mm. **(B)** Expression of glycolytic and OXPHOS markers (LDHA and COX7a1) at mRNA level. **(C–E)** qRT-PCR, western blot and immunofluorescence staining showed the expression levels of mitochondrial dynamic proteins of HIF-1α-modified hiPSCs. Scale bars, 20 mm. ^∗^*P* < 0.05, ^∗∗^*P* < 0.01, ^∗∗∗^*P* < 0.001 vs. HIF-1α NC hiPSCs. (Student’s *t* test). All data are representative of three independent experiments.

RETRACTED

Subsequently, the effects of HIF-1α modification on mitochondrial dynamics were assessed. The results showed that HIF-1α significantly disrupted the balance of mitochondrial dynamics. Notably, HIF-1α knockdown significantly enhanced the expression of the mitochondrial fusion protein MFN2, as demonstrated by qRT-PCR, western blot analysis, and immunofluorescence staining (Figures 1C–E).

### HIF-1α Regulates the NSC Differentiation Potential of hiPSCs *in vivo* and *in vitro*

As the results showed (Figure 1) that HIF-1α significantly inhibited the expression of MFN2 which has previously been reported to influence neural differentiation (Lee et al., 2012; Misko et al., 2012; Fang et al., 2016), we thus examined the effects of HIF-1α on the NSC differentiation potential of hiPSCs *in vitro* and *in vivo*. EB formation assays, simulating early human embryo development *in vivo* up to a point, were carried out. As described previously, HIF-1α knockdown could damage EB morphology and formation efficiency (Cui et al., 2020), indicating that HIF-1α knockdown significantly disturbed the spontaneous differentiation potential of hiPSCs. Then, EBs that were differentiated to the ninth day were adhered to Matrigel for 48 h, and the results of Mito tracker staining showed that the mitochondrial morphology of differentiated cells from HIF-1α OE hiPSCs tended to be fragmented, whereas differentiated cells from HIF-1α sh hiPSCs tended to be elongated (Figures 2A,B). Furthermore, the adherent differentiated culture medium was adjusted to NSC induction medium containing bFGF and EGF, and it was observed that HIF-1α knockdown significantly improved the spontaneous differentiation efficiency of NSCs, whereas HIF-1α overexpression significantly inhibited the spontaneous differentiation (Figure 2C). After the HIF-1α-modified hiPSCs were continuously cultured for 13 days in medium without factors to maintain pluripotency, HIF-1α sh hiPSCs spontaneously differentiated into neural-like cells, whereas the same phenomenon did not occur in HIF-1α OE hiPSCs (Figure 2D). This indicated that HIF-1α knockdown activated the neural differentiation signaling in hiPSCs under specific conditions. Subsequently, by using small molecule inhibitors that regulate neural differentiation signals to orient hiPSCs to NSCs, the results showed that HIF-1α knockdown promoted the directional differentiation potential of NSCs, whereas HIF-1α overexpression inhibited the directed differentiation potential (Figures 2E,F).

RETRACTED

**FIGURE 2:** Hypoxia-inducible factor 1α (HIF-1α) regulates the NSC differentiation potential of hiPSCs *in vivo* and *in vitro*. **(A,B)** Mito tracker staining showed the mitochondrial morphology of differentiated cells from HIF-1α-modified hiPSCs, red arrows, fragmented mitochondrias; asterisk, elongated mitochondria. Scale bars, 200 mm. **(C)** The cell morphology of the adherent EBs from HIF-1α-modified hiPSCs with NSC differentiation medium. Scale bars, 100 mm. **(D)** The cell morphology of HIF-1α-modified hiPSCs after continuously culturing for 13 days in medium without factors to maintain pluripotency. **(E,F)** Expression of Nanog and NSC markers (PAX6 and Nestin) by the directed inducing of small molecule inhibitors. Scale bars, 20 mm. **(G)** Immunohistochemical staining showed the expression levels of NSC markers (PAX6 and Nestin) of teratomas derived from HIF-1α-modified hiPSCs. Scale bar, 100 μm. ^∗^*P* < 0.05, ^∗∗^*P* < 0.01 vs. HIF-1α NC hiPSCs. (Student’s *t* test). All data of qRT-PCR are representative of three independent experiments.

To determine whether HIF-1α could regulate the neurodevelopment of hiPSCs *in vivo*, the teratoma formation assay was performed in the SCID mice. The immunohistochemical analysis results of NSC markers (PAX6 and Nestin) verified the effects of HIF-1α on the NSC differentiation and development of hiPSCs *in vivo* (Figure 2G). These results indicated that HIF-1α significantly influenced the neurodevelopment tendency of hiPSCs by regulating a series of metabolic programs and development-related genes.

### MFN2 Affects the NSC Differentiation Potential of hiPSCs by Regulating β-Catenin

Mitofusin2, a vital protein that regulates mitochondrial fusion and metabolism, also plays a pivotal role in neural differentiation and neurodegenerative diseases (Burte et al., 2015; Fang et al., 2016). To determine whether HIF-1α affects NSC differentiation by regulating MFN2 signaling, we investigated the effects of MFN2 on the NSC differentiation potential of hiPSCs. MFN2 overexpression and knockdown hiPSC cell lines (MFN2 OE and MFN2 sh hiPSCs, respectively) were established (Supplementary Figures 1A, 3A,B), and these had stable genetic properties *in vitro* (Supplementary Figure 1B). The results of qRT-PCR, western blot analysis, and AP activity detection showed that MFN2 has no significant effects on the pluripotency of hiPSC (Figure 3A,B and Supplementary Figure 1C). The results of CCK8 and clonogenic assays showed that MFN2 overexpression significantly reduced the self-renewal potential and clone formation efficiency of hiPSCs (Supplementary Figures 1D,E). Next, we tested the effects of MFN2 on mitochondrial characteristics and energy metabolism using the same methods described previously herein, and the results showed that MFN2 overexpression significantly reduced the ΔΨm of hiPSCs (Supplementary Figures 1F,G), and that MFN2 knockdown significantly decreased the degree of oxidative stress and intracellular ATP content in hiPSCs (Supplementary Figures 1H,K).

RETRACTED

**FIGURE 3:** Mitofusin2 (MFN2) affects the NSC differentiation potential of hiPSCs by regulating β-catenin. **(A,B)** Expression of MFN2, Nanog, and OCT4 (pluripotency markers) at mRNA and protein levels, and the bar chart showed the protein levels. β-actin and COX IV were used as control. **(C)** EBs morphology of MFN2-modified hiPSCs. Scale bars, 100 mm. **(D,E)** Bar graphs showed the EB formation efficiency **(D)** and the diameters of EBs **(E)**. **(F,G)** Mito tracker staining showed the mitochondrial morphology of differentiated cells from MFN2-modified hiPSCs, red arrows, fragmented mitochondria; asterisk, elongated mitochondria. Scale bars, 200 mm. **(H)** The cell morphology of the adherent EBs from MFN2-modified hiPSCs under NSC differentiation medium. Scale bars, 100 mm. **(I,J)** Expression of Nanog and NSC markers (PAX6 and Nestin) by directed inducing of small molecule inhibitors. Scale bars, 20 mm. **(K,L)** Western blot and immunofluorescence showed the expression levels of β-catenin in MFN2-modified hiPSCs. Scale bars, 20 mm. **(M,N)** Western blot and immunofluorescence showed the expression levels of β-catenin in HIF-1α-modified hiPSCs. Scale bars, 20 mm. ^∗^*P* < 0.05, ^∗∗^*P* < 0.01, ^∗∗∗^*P* < 0.001 vs. HIF-1α NC hiPSCs. (Student’s *t* test). All data of qRT-PCR are representative of three independent experiments.

To verify the effects of MFN2 modification on the NSC differentiation potential of hiPSCs, spontaneous EB differentiation assays were performed. The results showed that EBs formed by MFN2 OE hiPSCs were more irregular than those of MFN2 sh and MFN2 NC hiPSCs (Figure 3C), and that MFN2 overexpression significantly reduced EB formation efficiency and the diameter of hiPSCs (Figures 3D,E). Then, EBs differentiated to the ninth day were allowed to adhere, and the results of Mito tracker staining showed that the mitochondrial morphology of differentiated cells from MFN2 OE hiPSCs tended to be elongated, whereas differentiated cells from MFN2 sh hiPSCs tended to be fragmented (Figures 3F,G). The results of cell morphology and immunofluorescence with NSC markers of adherent EB cells showed that MFN2 overexpression significantly promoted the spontaneous differentiation of NSCs, while MFN2 knockdown significantly inhibited the spontaneous differentiation (Figure 3H and Supplementary Figure 2A). Meanwhile, we detected the effect of MFN2 modification on the NSC differentiation potential of hiPSCs through the NSC directed differentiation by small molecule inhibitor inducing, The results of qRT-PCR and immunofluorescence showed that MFN2 overexpression significantly increased the expression of NSC markers and the tendency of NSC differentiation (Figures 3I,J). In order to more accurately identify the effect of MFN2 modification on NSC differentiation and pluripotency during NSC differentiation, we examined the effect of MFN2 modification on the Nanog expression of hiPSCs 4 days before differentiation, and identified the expression of NSC markers at day 14 and 16 after differentiation. The results showed that MFN2 overexpression significantly accelerated the decrease of pluripotency levels of hiPSCs during differentiation, while MFN2 knockdown significantly delayed the decrease of pluripotency levels (Supplementary Figure 2B). The results of longer differentiation showed no significant change in the expression of NSC Markers (PAX6/Nestin) at day 12 and 16 (Supplementary Figure 2B). Therefore, the 12-day cycle was sufficient to complete the differentiation process of hiPSCs into NSC. Meanwhile, we also examined the changes in the expression of MFN2 at mRNA and protein levels during NSC differentiation. The results showed that the expression of MFN2 was significantly increased with the progression of NSC differentiation (Supplementary Figures 2C,D), and the mitochondrial fusion kinetics was significantly enhanced.

RETRACTED

In our previous study, excess mitochondrial fission impaired pluripotency, germ layer differentiation, and embryonic development potential by regulating the ubiquitin-mediated proteasomal degradation of β-catenin protein (Zhong et al., 2019). However, the mechanisms of whether HIF-1α-dependent energy metabolism could affect the NSC differentiation potential of hiPSCs by regulating mitochondrial fusion-mediated Wnt/β-catenin signaling remain elusive. The aforementioned results revealed that HIF-1α affected the NSC differentiation potential of hiPSCs via the regulation of MFN2 protein levels. The effects of HIF-1α/MFN2 on β-catenin expression were also investigated by western blot analysis and immunofluorescence staining, and the results showed that MFN2 significantly increased the level of β-catenin protein (Figures 3K,L), whereas HIF-1α, an upstream regulator of MFN2, significantly reduced the protein levels of β-catenin (Figures 3M,N). Therefore, the HIF-1α/MFN2/β-catenin axis plays a vital role in the pluripotency, self-renewal, and NSC differentiation potential of hiPSCs.

### MFN2 Reverses the Effects of HIF-1α Overexpression on the NSC Differentiation Potential of hiPSCs

Whether MFN2 could alleviate or rescue the effects on the NSC differentiation and β-catenin expression in hiPSCs was investigated. Based on HIF-1α overexpression, we further overexpressed MFN2 and established a stable cell line (DOE hiPSCs, Figures 4A,B). To further determine whether MFN2 could reverse the effects of HIF-1α overexpression on the NSC differentiation potential of hiPSCs, we performed EB spontaneous differentiation and small molecule inhibitor-induced NSC-directed differentiation assays on hiPSCs. The results showed that MFN2 overexpression significantly inhibited the EB status, formation ability and diameter of HIF-1α OE hiPSCs (Figures 4C–E), and qRT-PCR and immunofluorescence analysis showed that MFN2 overexpression significantly increased the efficiency and tendency of NSC spontaneous and directed differentiation of HIF-1α OE hiPSCs (Supplementary Figures 4F–H and Supplementary Figure 3). Furthermore, western blot analysis and immunofluorescence staining revealed that MFN2 overexpression could promote β-catenin expression in HIF-1α OE hiPSCs (Figures 4I,J). These results suggested that excessive mitochondrial fusion could reverse the effects of HIF-1α overexpression on self-renewal, mitochondrial metabolism, and β-catenin expression in hiPSCs, and could further improve the NSC differentiation potential of HIF-1α OE hiPSCs.

**FIGURE 4:** Mitofusin2 (MFN2) reverses the effects of HIF-1α overexpression on the NSC differentiation potential of hiPSCs. **(A,B)** Expression of MFN2, Nanog and OCT4 at mRNA and protein level. β-actin and COX IV were used as control. **(C)** EBs morphology of CON (hiPSCs), MFN2 OE, HIF-1α OE, and DOE hiPSCs. Scale bars, 100 mm. **(D,E)** Bar graphs showed the EB formation efficiency **(D)** and the diameters of EBs **(E)**. **(F)** The cell morphology of the adherent EBs from MFN2 and HIF-1α modified hiPSCs under NSC differentiation medium. Scale bars, 100 mm. **(G,H)** Expression of Nanog and NSC markers (PAX6 and Nestin) by directed inducing of small molecule inhibitors. Scale bars, 20 mm. **(I,J)** Western blot and immunofluorescence showed the expression levels of β-catenin in CON, MFN2 OE, HIF-1α OE, and DOE hiPSCs. Scale bars, 20 mm. ^∗^*P* < 0.05, ^∗∗^*P* < 0.01, ^∗∗∗^*P* < 0.001 vs. CON or MFN2 OE hiPSCs. ^#^*p* < 0.05, ^##^*p* < 0.01 vs. HIF-1α OE hiPSCs (Student’s *t* test). All data of qRT-PCR are representative of three independent experiments.

RETRACTED

### Wnt/β-Catenin Signaling Inhibition Reverses the Effects of HIF-1α Knockdown on the NSC Differentiation Potential of hiPSCs

To further determine whether Wnt/β-catenin signaling inhibition could reverse the effects of HIF-1α knockdown on the NSC differentiation potential of hiPSCs. We identified the effects of different concentrations of Wnt/β-catenin signaling inhibitor XAV939 on the expression of Wnt/β-catenin-related signaling proteins (WNT3a, WNT5a, GSK-3β, β-catenin, Cyclin D1, Axin1, and DKK1) in hiPSCs, and the results showed that XAV939 at a concentration of 1 μM could significantly inhibit the expression of Wnt/β-catenin-related signaling proteins (WNT3a, WNT5a, GSK-3β, and β-catenin) in hiPSCs after 6 days of culturing (Figure 5A). In order to detect the effects of Wnt signaling pathway inhibitor XAV939 on the pluripotency and self-renewal potential of hiPSCs, the results of CCK8 assay, Western blot assay and clone formation assay showed that 1 μM XAV939 significantly inhibited the self-renewal, pluripotency and clone formation ability of hiPSCs (Supplementary Figures 4A–E). These results indicated that Wnt signaling pathway plays an extremely important role in the biological characteristics of hiPSCs. Previous research has shown that self-renewal of stem cells is maintained in the absence of β-catenin (Lyashenko et al., 2011). Hence, other key proteins in the Wnt signaling pathway may play a pivotal role in stem cell self-renewal and maintenance of pluripotency. Meanwhile, we detected the effect of HIF-1α modification on the expression of Wnt/β-catenin-related signaling proteins. The results showed that HIF-1α knockdown significantly increased the expression of Wnt/β-catenin-related signaling proteins, while HIF-1α overexpression significantly inhibited Wnt/β-catenin signaling (Figure 5B). Furthermore, we performed EB spontaneous differentiation and small molecule inhibitor-induced NSC-directed differentiation assays on hiPSCs. The results showed that XAV939 significantly affected the EB status, formation ability and diameter of HIF-1α NC and HIF-1α sh hiPSCs to some extent (Figures 5C–E), and qRT-PCR and immunofluorescence analysis showed that XAV939 significantly inhibited and reversed the efficiency and tendency of NSC spontaneous and directed differentiation of HIF-1α sh hiPSCs (Figures 5F–H and Supplementary Figure 4F).

**FIGURE 5:** Wnt/β-catenin signaling inhibition reverses the effects of HIF-1α knockdown on the NSC differentiation potential of hiPSCs. **(A)** Effects of different concentrations of XAV939 (Wnt/β-catenin signaling inhibitor) on the expression of Wnt/β-catenin signaling-related proteins in hiPSCs. β-actin was used as control. **(B)** Effects of HIF-1α on the expression of Wnt/β-catenin signaling-related proteins in hiPSCs. β-actin was used as control. **(C)** EBs morphology of HIF-1α NC and HIF-1α sh hiPSCs with 1 μM XAV939. HIF-1α NC and HIF-1α sh hiPSCs were used as control for HIF-1α NC and HIF-1α sh hiPSCs with 1 μM XAV939. Scale bars, 100 mm. **(D,E)** Bar graphs showed the EB formation efficiency **(D)** and the diameters of EBs **(E)**. **(F)** The cell morphology of the adherent EBs from HIF-1α NC/sh hiPSCs and HIF-1α NC/sh hiPSCs with 1 μM XAV939 under NSC differentiation medium. Scale bars, 100 mm. **(G,H)** Expression of Nanog and NSC markers (PAX6 and Nestin) by directed inducing of small molecule inhibitors. Scale bars, 20 mm. *P < 0.05, **P < 0.01, ***P < 0.001 vs. CON or HIF-1α NC hiPSCs. ###*p* < 0.001 vs. HIF-1α sh hiPSCs (Student’s *t* test). All data of qRT-PCR are representative of three independent experiments.

RETRACTED

## Discussion

Hypoxia-inducible factor 1α, a regulator of glycolytic metabolism, plays a key role in inducing the pluripotency and directional differentiation of stem cells after initiating the conversion of early glycolytic metabolic programs (Semenza, 2012). Hypoxia significantly increases the transcription of target genes of HIF-1α, such as *LDHA*, *PDK1*, *BNIP3*, *COX4-2*, and *LON*, which play important roles in regulating mitochondrial metabolism and cell performance (Prigione et al., 2014). In this study, we showed that HIF-1α knockdown significantly inhibited the mitochondrial membrane potential of hiPSCs. Additionally, HIF-1α knockdown significantly increased intracellular ROS production, thereby enhancing the oxidative stress response in hiPSCs. These mitochondrial changes caused by HIF-1α knockdown likely contribute to the significant inhibition of hiPSC pluripotency and self-renewal potential. Previous studies have shown that the different metabolic patterns in stem cells are closely related to reprogramming and cell fate decisions (Gu et al., 2016). The loss of HIF-1α function seriously hinders the reprogramming efficiency of somatic cells, and the closely related metabolic regulatory factors of HIF-1α, including pyruvate dehydrogenase kinase 3 (PDK3) and pyruvate kinase isoform M2 (PKM2), significantly increase the reprogramming efficiency by improving glycolysis activity. At the same time, small molecule-induced HIF-1α activation significantly changes the fate of stem cells (Kim et al., 2006; Zhu et al., 2010; Prigione et al., 2011). Our results showed that HIF-1α overexpression significantly increased the glycolytic activity of hiPSCs, whereas HIF-1α knockdown significantly increased mitochondrial OXPHOS activity, suggesting that HIF-1α affected the conversion of metabolic patterns in hiPSCs. The results of the NSC differentiation and development assays showed that HIF-1α knockdown significantly improved the NSC differentiation tendency and developmental potential of hiPSCs, indicating that HIF-1α plays a key role in determining the differentiated fate of hiPSCs. Therefore, a comprehensive understanding of the underlying mechanisms that affect HIF-1α biology in hiPSCs will provide crucial insights into stem cell biology and regenerative medicine.

RETRACTED

The balance of mitochondrial dynamics that depend on mitochondrial fusion and fission is not vital for the survival of stem cells (Lisowski et al., 2018), but it is essential for pluripotency, reprogramming, and normal embryonic development (Chen and Chan, 2010; Xu et al., 2013). Notably, mitochondrial fusion disorders can result in various metabolic and neurodegenerative diseases (Züchner et al., 2004; Misko et al., 2012). In view of the importance of MFN2 in mitochondrial performance and neurodevelopment, this study identified that MFN2 overexpression significantly decreased the self-renewal potential and mitochondrial metabolism of hiPSCs, and it significantly increased the NSC differentiation potential of hiPSCs. Whereas, MFN2 knockdown increased mitochondrial membrane potential, and reduced intracellular oxidative stress levels, which further inhibits the NSC differentiation and development potential of hiPSCs. MFN2 could reverse the effects of HIF-1α overexpression on self-renewal, mitochondrial performance, and the NSC differentiation potential of hiPSCs. Despite the importance of mitochondrial fusion for cell fate determination, MFN2 is more essential than mitofusin1 in maintaining embryonic development and neural differentiation (Lee et al., 2012; Pham et al., 2012). Moreover, mitochondrial dynamics could regulate epigenetic modification and affect cell life processes such as autophagy and aging (Hu and Liu, 2014; Xiong et al., 2014). Histone deacetylase Sirt4 is closely related to aging, and similar to MFN2 functioning in mitophagy, Sirt4 could inhibit cellular autophagy by promoting mitochondrial fusion (Lang et al., 2017). Our previous studies have shown that HIF-1α-dependent mitochondrial energy metabolism affected the differentiation and development potential of hiPSCs via regulating histone epigenetic modifications (Cui et al., 2020). The balance of mitochondrial dynamics regulated by key metabolism genes and epigenetic modifications and affects hiPSC autophagy and apoptosis is an important field that requires further investigation; especially, it has important prospects for improving the metabolic disorders related to premature aging.

RETRACTED

Based on accumulating evidence, Wnt/β-catenin signaling plays a key role in maintaining the pluripotency of PSCs and facilitates cell reprogramming (Miki et al., 2011). Specifically, β-catenin has been reported to be a functional factor that initiates the differentiation of PSCs (Kelly et al., 2011; Liu et al., 2017). Importantly, β-catenin knockout leads to embryonic lethality due to disrupted mesoderm formation and neural differentiation capacity, which also interferes with cell metabolism pathway regulation (Lyashenko et al., 2011). Therefore, the maintenance of Wnt/β-catenin signal activity plays a vital role in the neural development and metabolism of PSCs. MFN2, as a key mitochondrial and metabolism-related protein, plays pivotal roles in maintaining the stable metabolism, pluripotency and neuroectodermal differentiation and development of PSCs. Therefore, whether MFN2 influence Wnt/β-catenin signaling by regulating energy metabolism related pathways, thus affecting the neural differentiation potential of PSCs is worthy of further discussion. For the future study, it is necessary to verify whether MFN2-regulated metabolic pathway inhibitors or small molecules could significantly affect Wnt/β-catenin signal and neural differentiation, which will further broaden and strengthen our understanding of the mechanism of mitochondrial dynamics affecting stem cell differentiation and development. Calmodulin is considered a key effector molecule of the non-classical Wnt signaling pathway (Bengoa-Vergniory and Kypta, 2015). Moreover, our previous studies have shown that the balance of mitochondrial dynamics affects the developmental potential of PSCs by regulating CaMKII-dependent β-catenin degradation (Zhong et al., 2019). The present study revealed that HIF-1α significantly affected the NSC differentiation and developmental potential of hiPSCs via mitochondrial fusion protein MFN2-mediated β-catenin signaling. Our findings broaden our understanding of the effects of metabolic regulatory proteins, mitochondrial dynamics, and the non-canonical Wnt pathway on neural differentiation and the development of hiPSCs.

Nevertheless, whereas the role of mitochondrial metabolism and dynamics in the pluripotency and differentiation potential of PSCs has attracted increasing attention, very little is known about the underlying molecular mechanisms involved in this process. Our results provide a novel perspective, in that HIF-1α could affect the NSC differentiation potential of hiPSCs by regulating mitochondrial fusion-mediated Wnt/β-catenin signaling (Figure 6). This contributes to our understanding of the NSC differentiation regulation of hiPSCs, and provides molecular insight that could be useful for the development of novel neurodegenerative disease treatment strategies. However, the molecular mechanism of how HIF-1α regulates mitochondrial dynamics mediated NSC differentiation through nuclear transcriptional interactions is still missing, and the influence mechanism of HIF-1α on the differentiation of terminal functional nerve cells (neurons, oligodendrocytes, and astrocytes) still needs to be further verified. Whether mitochondrial dynamic proteins could affect nerve cell differentiation through interaction is an important direction.

RETRACTED

**FIGURE 6:** Hypoxia-inducible factor 1α (HIF-1α)/MFN2/β-catenin axis is required for the NSC differentiation of hiPSCs. HIF-1α-dependent mitochondrial energy metabolism significantly affected pluripotency and the self-renewal potential of hiPSCs. HIF-1α could significantly affect the NSC differentiation potential of hiPSCs by regulating MFN2-mediated β-catenin. Meanwhile, MFN2 could reverse the effects of HIF-1α knockdown on self-renewal, mitochondrial energy metabolism, NSC differentiation potential and β-catenin expression of hiPSCs.

## Data Availability Statement

The raw data supporting the conclusions of this article will be made available by the authors, without undue reservation.

## Ethics Statement

The animal study was reviewed and approved by Peking University Shenzhen Hospital.

## Author Contributions

PC, PZ, and LY designed and performed the experiments, analyzed the data, and wrote the manuscript. LW, XG, GC, YZ, ML, and XZ performed the majority of experiments. XL and YY conceived and supervised this study. ZY provided the funding support and also supervised this work. All the authors read and approved the manuscript.

## Conflict of Interest

The authors declare that the research was conducted in the absence of any commercial or financial relationships that could be construed as a potential conflict of interest.
